RETRACTED

# The Polyherbal Wattana Formula Displays Anti-Amyloidogenic Properties by Increasing α-Secretase Activities

**DOI:** 10.1371/journal.pone.0170360

**Published:** 2017-01-20

**Authors:** Htut Htut Htoo, Suveerawan Limsuvan, Onusa Thamsermsang, Jean-François Hernandez, Frédéric Checler, Piyarat Govitrapong, Narawut Pakaprot, Pravit Akarasereenont, Bruno Vincent

**Affiliations:** 1 Institute of Molecular Biosciences, Mahidol University, Nakhon Pathom, Thailand; 2 Center of Applied Thai Traditional Medicine, Faculty of Medicine Siriraj Hospital, Mahidol University, Bangkok, Thailand; 3 Institut des Biomolécules Max Mousseron, UMR5247 CNRS/Université de Montpellier/ENSCM, Faculté de Pharmacie, Montpellier, France; 4 Université Côte d’Azur, INSERM, CNRS, IPMC, Laboratory of excellence DistALZ, Sophia-Antipolis, Valbonne, France; 5 Center for Neuroscience and Department of Pharmacology, Faculty of Science, Mahidol University, Bangkok, Thailand; 6 Research Center for Neuroscience, Institute of Molecular Biosciences, Mahidol University, Nakhon Pathom, Thailand; 7 Department of Physiology, Faculty of Medicine Siriraj Hospital, Mahidol University, Bangkok, Thailand; 8 Department of Pharmacology, Faculty of Medicine Siriraj Hospital, Mahidol University, Bangkok, Thailand; 9 Centre National de la Recherche Scientifique, Paris, France; Torrey Pines Institute for Molecular Studies, UNITED STATES

## Abstract

Alzheimer’s disease is characterized by the deposition of insoluble amyloid-β peptides produced from the β-amyloid precursor protein (βAPP). Because α-secretase cleavage by ADAM10 and ADAM17 takes place in the middle of Aβ, its activation is considered as a promising anti-AD therapeutic track. Here we establish that the polyherbal Wattana formula (WNF) stimulates sAPPα production in cells of neuronal and non-neuronal origins through an increase of both ADAM10 and ADAM17 catalytic activities with no modification of BACE1 activity and expression. This effect is blocked by specific inhibition or genetic depletion of these disintegrins and we show that WNF up-regulates ADAM10 transcription and ADAM17 maturation. In addition, WNF reduces Aβ40 and Aβ42 generation in human cell lines. Altogether, WNF presents all the characteristics of a potent preventive anti-Alzheimer formula. Importantly, this natural recipe, currently prescribed to patients for the treatment of other symptoms without any secondary effect, can be tested immediately for further clinical studies.

## Introduction

Alzheimer’s disease (AD) is a progressive and yet incurable neurodegenerative disorder affecting the elderly. This syndrome, at its early stage, is characterized by mild memory loss before evolving to a severe decline of cognitive functions and ultimately leading to dementia and death. At the molecular level, proteolysis of the β-amyloid precursor protein (βAPP) by enzymes called “secretase” is a central event since it determines both the production rate and the nature of the amyloid peptide (Aβ) [1], the main component of the extracellular senile plaques formed in the brain of affected individuals. On one hand, the so-called “amyloidogenic” pathway leading to Aβ production is a two-step mechanism along which the β-secretase BACE1 (Beta-site APP-Cleaving Enzyme 1) first generates its N-terminal extremity before Aβ generation is completed by the heterotetrameric γ-secretase complex that liberates the C-terminal end of the peptides. On the other hand, there exists an alternative “non amyloidogenic” route of βAPP processing that is mainly performed by ADAM10 and ADAM17, two members of the ADAM (A Disintegrin And Metalloprotease) family. Importantly, this cleavage of βAPP triggers two beneficial effects regarding AD since it is not only taking place in the middle of the Aβ sequence, thereby preventing its production, but also gives rise to a large sAPPα secreted fragment that displays neuroprotective, neurotrophic, memory-enhancing and neurogenesis-stimulating properties [2–6]. For these reasons, sAPPα is largely considered as a key positive factor in terms of AD. On a therapeutic point of view, besides the promising but yet unsuccessful vaccination approach, numerous studies aimed at inhibiting the amyloidogenic β- and γ-secretases or activating the non-amyloidogenic α-secretases were conducted during the past years [7, 8]. However, acute pharmacological modulation of α-secretases, that are implicated in a wide range of AD-unrelated and important physiological processes, is hardly conceivable as an anti-AD therapy in humans since it would likely trigger some serious side effects, thereby impairing the therapeutic success of such molecules [9]. It has been proposed that an alternative to pharmaceutical therapies could be to regulate these proteases through the regular consumption of natural compounds (nutrients, plant constituents or herbal extracts) that would operate in a mild but chronic manner throughout life (for review see [10]).

RETRACTED

The Thai Wattana formula (WNF), a polyherbal mixture, has been traditionally used for health prevention and nourishment from age-related problems like loss of appetite, weakness, digestion and gastrointestinal problems. This formula is composed of 15 medicinal plants: *Aegle marmelos* (L.) Corrêa (Bael fruit), *Boesenbergia rotunda* (L.) Mansf. (Krachai), *Cinnamomum ilicioides* A. Chev. (Ka Thon), *Cladogynosorientalis* Zipp. ex Span. (Chetta Phang Khi), *Cryptolepis dubia* (Burm.f.) M.R.Almeida (Soften tendons), *Cyperusrotundus* L. (Nutgrass), *Derris scandens* (Roxb.) Benth. (Jewel Vine), *Putrangiva roxburghii* Wall. (Ma Kham Kai), a gum of *Ferula assafoetida* L. (Asafetida), *Ligusticum sinense* Oliv. (Kot Hua Bua), *Mallotusrepandus* (Willd.) Mull.Arg. (Kho Khlan/Fishberry), *Piper nigrum* L. (White Pepper), *Aucklandia lappa* DC. (Costus), *Terminalia chebula* Retz. (Myrobalans) and *Tinospora crispa* (L.) Hook.f. (Bora Phet) [11]. It is generally prescribed as an appetite stimulant and for health improvement and promotion. Moreover, it has recently been tested for its ability to control the immunomodulatory activity of natural killer and monocyte-derived dendritic cells, osteoarthritis and gastric emptying rate (GER) [12–15]. Finally, it has been shown to convey protection against ultraviolet A-induced melanogenesis through an antioxidant/redox mechanism [11]. Because this formula was also proposed to have some anti-aging properties, we examined its possible beneficial effect in an AD-related context. Here we demonstrate that WNF promotes the non amyloidogenic α-secretase processing of βAPP in neuronal and non-neuronal cells through the activation of ADAM10 and ADAM17 catalytic activities without interfering with β-secretase (BACE1) activity and expression. We also show that WNF regulates these two disintegrins through distinct transcriptional and post-transcriptional mechanisms. Finally, we establish that WNF is able to reduce amyloid peptides production in cells *in vitro*.

## Materials and methods

### Materials

DMEM, Opti-MEM, geneticin, fetal bovine serum (FBS) and lipofectamine 2000 were from Invitrogen (Carlsbad, CA, USA). Penicillin-streptomycin mix was from PAA. Tris and Glycine were from Vivantis (Selangor Darul Ehsan, Malaysia). PDBu, poly-D-lysine, GI254023X and dimethyl sulfoxide were from Sigma (St Louis, MO, USA). Skim milk powder was from HiMedia (Mumbai, India). Ammonium persulphate was from GE Health care (Pisataway, NJ, USA). The chemiluminescence HRP substrate was from Millipore (Bedford, MA, USA). SDS was from Amaresco (Solon, OH, USA). O-Phenanthroline and TAPI-0 were from Calbiochem (San Diego, CA, USA).

### Preparation and analysis of WNF

The sources of all herbal components came from the wild stretching from the Central and the Northeastern parts of Thailand by contact suppliers who collected and sold the crude herbs to the Center of Applied Thai Traditional Medicine where the origin of each herb was recorded. All the production procedures were then supported by the Manufacturing Unit of Herbal Medicines and products, Center of Applied Thai Traditional Medicine (CATTM), Faculty of Medicine Siriraj Hospital (Bangkok) and were operated under Good Manufacturing Practice (GMP) certification. Briefly, individual herbs were first authenticated by experts, including certified pharmacognosists of the Center of applied Thai traditional medicine. All of raw materials were washed with de-ionized water (DI), dried by hot-air oven and then grinded, sieved and packed in laminated vacuum packaging bags. The polyherbal formula powder is then obtained by extraction of equal amount of each herb (weight/weight) with an 80% ethanol solution at a final concentration of 100mg/ml, filtered through cotton wool and subsequently centrifuged at 10,000xg for 10 min. The supernatant was evaporated and lyophilized to obtain freeze-dried powder and stored in amber bottle at 25°C in desiccators. The physical properties, the heavy metal and microbial contamination of formula were assessed before any experiment is performed. In addition, the chemical assessments of the formula were verified using Thin Layer Chromatography (TLC) and Ultra Performance Liquid Chromatography (UPLC) as previously described [11]. WNF was freshly prepared before experimental use on cell lines as a 10mg/ml stock solution in 50% DMSO.

RETRACTED

### Cell lines, transfections and in vitro treatments

Human HEK293 cells and mouse embryonic fibroblasts (MEFs) were cultured at 37°C, 5% CO_2_ in DMEM supplemented with 10% FBS, penicillin (100U/ml) and streptomycin (50mg/ml). HEK293 cells stably overexpressing human βAPPwt_751_, human ADAM10, mouse ADAM17 or 1D4-tagged human BACE1 were obtained and maintained as previously described [16–18]. Mouse neuroblastoma N2a cells stably overexpressing human wild-type neuronal βAPP_695_ [19] were cultured at 37°C, 5% CO_2_ in 50% DMEM, 50% Opti-MEM, supplemented with 5% FBS, antibiotics and geneticin (0.25g/l). MEFs derived from ADAM10^-/-^ or ADAM17^-/-^ mice (as well as wild-type controls) were previously described [20, 21]. Human SH-SY5Y neuroblastoma cells were grown at 37°C, 5% CO_2_ in 50%DMEM/50%F12 containing 10% FBS, glutaMAX (2mM), non-essential amino-acids (0.05%) and antibiotics. Transient overexpression of human wild-type βAPP_751_ in MEFs, HEK293 and SH-SY5Y cells was carried out with lipofectamine 2000. WNF was prepared as a 10mg/ml solution by adding 1 ml of 50% DMSO/50% H_2_O to 10mg of desiccated pellet and used for the 100μg/ml treatments. Serial dilutions were performed for lower concentrations. For all conditions (including non-treated controls), DMSO was adjusted to 0.5%.

### sAPPα secretion and western blot analysis

Secretion and detection of sAPPα in HEK293, N2a, SH-SY5Y and MEFs with the human-specific monoclonal DE2B4 antibody (dilution 1/500, Santa Cruz Biotechnology Inc., Santa Cruz, CA, USA) has been previously described [22]. Cells were collected with phosphate-buffered saline (PBS)-EDTA and resuspended in 80 to 150 μl of lysis buffer (10mM Tris/HCl, pH 7.5, 150mM NaCl, 0.5% triton X-100, 0.5% deoxycholate, 5mM EDTA). Protein concentrations were determined by the Bradford method [23] and proteins were separated by SDS-PAGE on 8% (βAPP, calnexin and ADAM17) or 10% Tris/glycine (ADAM10, BACE1, Golgi 58K protein and β-actin), or 16.5% Tris/tricine gels (C83). Proteins were transferred onto nitrocellulose membranes (45 to 120min according to protein size, 100V), blocked for 1h in 5% non-fat milk and incubated overnight at 4°C with primary antibodies directed against βAPP/C83 (dilution 1/4000, polyclonal A8717, Sigma), ADAM10 (dilution 1/500, polyclonal AB19026, Millipore, Bedford, MA, USA), ADAM17 (dilution 1/1000, polyclonal AB19027, Millipore), BACE1 (dilution 1/1000, monoclonal EPR3956, Abcam, Cambridge, UK), calnexin (dilution 1/1000, monoclonal 610523, BD Biosciences, Singapore), Golgi 58K protein (dilution 1/2000, monoclonal G2404, Sigma) or β-actin (dilution 1/5000, monoclonal 13E5, Cell Signaling, Beverly, MA, USA). Bound antibodies were detected using goat anti-mouse (dilution 1/3000, polyclonal 7076, Cell Signaling) or goat anti-rabbit peroxidase-conjugated antibody (dilution 1/3000, polyclonal 7074, Cell Signaling). Immunological complexes were revealed using ECL methods (Immobilon Western Chemiluminescence HRP substrate) and detected using an automatic medical X-ray processor (Kodak, Rochester, NY, USA). Bands densitometries were measured with the ImageJ software and normalized using β-actin as internal standard.

RETRACTED

### α-secretase fluorimetric assay on intact cells

Wild-type, ADAM10^-/-^ or ADAM17^-/-^ MEFs as well as HEK293 cells overexpressing ADAM10 or ADAM17 were cultured in 35mm-dishes coated with polylysine (10μg/ml) until cells reached 80% confluence. Cells were treated in duplicate without (control) or with WNF (100μg/ml) for 16 hours at 37°C in 1ml of DMEM containing 1% FBS. After this treatment period, the PKC activator phorbol 12, 13-dibutyrate (PDBu) (1μM, wild-type/ADAM17^-/-^ MEFs and ADAM17-overexpressing HEK293 cells) was added for two hours. Duplicates were then incubated for 30 min at 37°C in the absence or in the presence of o-phenanthroline (general metalloprotease inhibitor, 100μM), GI254023X (ADAM10-specific inhibitor, 10μM), or TAPI-O (ADAM17-specific inhibitor, 10μM) in 1.5ml of PBS. Then, the α-secretase-specific JMV2770 substrate (10μM) [24] was directly added into the media and cells were maintained at 37°C. At each time point, 100μl of media were removed and the α-secretase-specific activity corresponding to the o-phenanthroline-, GI254023X- or TAPI-O-sensitive fluorescence was recorded in black 96-well plates at 320nm and 420nm excitation and emission wavelengths respectively.

RETRACTED

### β-secretase fluorimetric assay on cell homogenates

HEK293 cells stably overexpressing 1D4-BACE1 were cultured in 35mm-dishes until they reach 80% confluence, treated without (control) or with WNF (100μg/ml) for 16 hours at 37°C in DMEM containing 1% FBS and assayed for their β-secretase activity as previously described [16]. Briefly, cells were collected, lysed with Tris 10mM pH 7.5, homogenized and kept on ice. Samples were assayed for their protein contents with the Bradford method and all adjusted to a 3μg/μl concentration. Thirty μg of each samples (10μl) diluted in 10mM sodium acetate buffer pH 4.5 were incubated for 30 min at 37°C in black 96-well plates (in a final volume of 100μl) in the absence (triplicate) or in the presence (triplicate) of the β-secretase specific inhibitor JMV1197. Then, the β-secretase-specific JMV2236 substrate (10μM) was added to all samples and the β-secretase-specific activity corresponds to the JMV1197-sensitive fluorescence recorded at each time point at 320nm and 420nm excitation and emission wavelengths respectively.

### Real-time quantitative polymerase chain reaction (q-PCR)

Following treatments (36 hours), total RNA was extracted and purified with the PureLink RNA mini kit (Ambion, Life Technologies, Austin, TX, USA). Real-time PCR was performed with 100ng of total RNA using the QuantiFast SYBR Green RT-PCR kit (Qiagen, Singapore) detector system (Eppendorf Mastercycler ep RealPlex) and the SYBR Green detection protocol. The 2x QuantiFast SYBR Green RT-PCR master mix, QuantiFast RT mix, QuantiTectPrimer Assay and template RNA were mixed and the reaction volume was adjusted to 25μl using RNase-free water. The specific primers were designed and purchased from Qiagen. Each primer is a 10x QuantiTect Primer Assay containing a mix of forward and reverse primers for specific targets: Hs_ADAM10_1_SG (QT00032641, human ADAM10), Hs_ADAM17_1_SG (QT00055580, human ADAM17) and Hs_GAPDH_1_SG (QT00079247, human GAPDH).

### Sucrose gradient sub cellular fractionation

Wild-type HEK293 cells cultured in 100mm-dishes were incubated for 16 hours without (control) or with WNF (100μg/ml) in DMEM/1% FBS. Cells were then homogenized with a dounce homogenizer in 0.25M sucrose prepared in 10mM Tris-HCl (pH 7.4) and containing 1mM Mg(AcO)_2_. Equal amounts of protein were loaded at the top of a step gradient, centrifuged and fractions (1ml) were collected from top to bottom of each gradient. Proteins in fractions were precipitated overnight at 4°C with methanol (4 volumes) and calnexin, Golgi 58K protein, ADAM10 and ADAM17 immunoreactivities were analyzed by western blot as described above.

RETRACTED

### Measurement of human Aβ production

HEK293 and SH-SY5Y neuroblastoma cells were transiently transfected with the human wild-type βAPP_751_ cDNA for 36 hours and incubated without (control) or with various WNF concentrations during the last 16 hours (in 1ml of DMEM/FBS1%). Aβ40 and Aβ42 levels were then detected in the secretion media (50μl) using sandwich ELISA kits detecting human Aβ40 (khb3482) and human Aβ42 (khb3442) respectively (Invitrogen) following manufacturer’s recommendations. Aβ levels (pg/ml) were obtained by reading absorbance at 450nm with a spectrophotometer and values were then normalized with βAPP and β-actin.

### Statistical analysis

Statistical analyses were performed with the Prism software (GraphPad, San Diego, USA) using the unpaired t test for pair wise comparisons. All results were expressed as means ± SEM and the *p* values equal to or less than 0.05 were considered significant.

## Results

We first evaluated the effect of WNF on the non-amyloidogenic α-secretase processing of βAPP by cultured human HEK293 cells overexpressing βAPP_751_ and showed that concentrations from 1 up to 100μg/ml dose-dependently increase the secretion of sAPPα as well as the production of the α-secretase-derived C-terminal counterpart (C83 fragment) without modifying βAPP immunoreactivity (Fig 1A), thereby indicating that WNF most likely up-regulates the α-secretase processing of βAPP rather than βAPP expression. Considering the well-established roles of ADAM10 and ADAM17 in the constitutive and PKC-regulated α-secretase processing of βAPP respectively [25], we tested the effects of the ADAM10-specific inhibitor GI254023X as well as the ADAM17-specific inhibitor TAPI-O on the WNF-induced sAPPα production. The results showed that GI254023X and TAPI-O respectively prevent the constitutive (Fig 1B) and PDBu-stimulated (Fig 1C) WNF-dependent sAPPα secretion in βAPP-overexpressing HEK293 cells. Because these experiments were conducted in HEK293 cells artificially overexpressing high amounts of the βAPP protein, we then wanted to determine whether WNF was able to generate similar effects in the same cell line producing endogenous levels of βAPP. Indeed, WNF dose-dependently and significantly promotes sAPPα release without interfering with βAPP protein levels in wild-type HEK293 cells (Fig 1D).

**Fig 1:** WNF stimulates sAPPα production in human HEK293 cells. (A) Cultured βAPP_751_-HEK293 cells were incubated without (control) or with the indicated concentrations of WNF (in 1ml DMEM/1% FBS) for 16 hours at 37°C. After secretion for 1 hour (in 1ml serum-free DMEM), media and cell lysates were collected and sAPPα (n = 8), βAPP (n = 8), C83 (n = 6) and β-actin were analyzed by Western blot. (B, C) Cells were treated with the indicated WNF concentrations for 16 hours, subsequently stimulated (+) or not (-) for 2 hours with PDBu (1μM) (C) and then incubated for 30 min in the absence (-) or in the presence (+) of GI254023X (10μM) (B) or TAPI-0 (10μM) (C). Measure of sAPPα secretion and detection were performed as in (A). (D) Wild-type HEK293 cells were treated as in (A) and allowed to secrete for 5 hours before sAPPα (medium, n = 4) as well as βAPP (n = 4) and β-actin (lysate) were analyzed by Western blot. *p<0.05; **p<0.02; ***p<0.001; #p<0.0001; ns, non-statistically different. Immunoblots illustrate representative gels and histograms correspond to the statistical analysis for all experiments. All bars correspond to the densitometry analyses (βAPP and C83 being normalized with β-actin), are expressed as a percentage of control (white bars, non treated cells) taken as 100 and are the means ± SE of the indicated number of independent experiments. Black lines in (B) and (C) indicate when lanes from the same original gels were spliced for better clarity.

RETRACTED

We then validated these data in cells of neuronal origin and carried out similar experiments with cultured mouse N2a neuroblastoma cells stably overexpressing the neuron-specific βAPP_695_ isoform. As observed in HEK293 cells, WNF stimulates the secretion of sAPPα in a dose-dependent manner without altering βAPP levels (Fig 2A). We then wanted to ascertain that the formula conveys similar effects on the endogenous α-secretase processing of βAPP and established that WNF significantly increases endogenous sAPPα secretion in a dose-dependent manner in human SH-SY5Y neuroblastoma cells (Fig 2B).

**Fig 2:** WNF promotes sAPPα production in mouse and human neuroblastoma cell lines. Cultured βAPP_695_-N2a mouse cells (A) or wild-type SH-SY5Y human cells (B) were incubated without (control) or with the indicated concentrations of WNF (in 1ml DMEM/1% FBS) for 16 hours at 37°C. After secretion for 1 hour (A) or 3 hours (B) (in 1ml serum-free DMEM), media and cell lysates were collected and sAPPα, βAPP and β-actin were analyzed by Western blot. Immunoblots illustrate representative gels and histograms correspond to the statistical analysis for all experiments. All bars correspond to the densitometry analyses (βAPP being normalized with β-actin), are expressed as a percentage of control (white bars, non treated cells) taken as 100 and are the means ± SE of 8 (A) or 6 (B) independent experiments. *p<0.05; **p<0.02; ***p<0.002; #p<0.0001; ns, non-statistically different.

RETRACTED

We then used a specific and reliable α-secretase-specific fluorimetric assay [24] to investigate the effect of WNF (100μg/ml) on ADAM10 and ADAM17 catalytic activities. We observed that WNF triggers a significant increase of both the constitutive (ADAM10-expressing HEK293 cells) (Fig 3A) and PKC-regulated (PDBu-treated ADAM17 expressing cells) (Fig 3B) o-phenanthroline-sensitive JMV2770-hydrolyzing activities. Similar experiments performed using GI254023X (ADAM10-specific) and TAPI-O (ADAM17-specific) inhibitors indicated that WNF significantly triggers both GI254023X- (Fig 3C) and TAPI-O-sensitive (Fig 3D) JMV2770 degradation and confirmed that WNF indeed targets ADAM10 and ADAM17. We also evaluated the impact of WNF treatment on the amyloidogenic BACE1 catalytic activity by means of a specific fluorimetric assay [16]. As shown in Fig 3E, WNF applied at a concentration of 100μg/ml did not affect the JMV1197-sensitive JMV2236 degradation in BACE1-overexpressing HEK2983 cells. Moreover, WNF treatments did not modify endogenous BACE1 immunoreactivity in wild-type HEK293 cells (Fig 3F).

**Fig 3:** WNF increases α-secretase catalytic activities in HEK293 cells without interfering with BACE1 activity and expression. (A-D) Cultured ADAM10-HEK293 (A, C) or ADAM17-HEK293 (B, D) cells were treated in duplicate with (black circles) or without (control, white circles) WNF (100μg/ml in DMEM/1% FBS) for 16 hours at 37°C. Cells in (B) and (D) were then treated with PDBu (1μM) for 2 hours. Duplicates were subsequently incubated in PBS with or without o-phenanthroline (100μM) (A-B), GI254023X (10μM) (C) or Tap-I (10μM) (D) for 30 min. JMV2770 (10μM) was then added, media (100μl) were collected at the indicated time points and fluorescence was recorded. Values in curves represent the means ± SE of the specific (inhibitor-sensitive) fluorescence recorded during independent experiments (n = 4). For histograms, values in black bars are expressed as the percent of control (white bars) at each time and are the means ± SE of 4 independent experiments. *p<0.002; **p<0.0001. (E) Cultured 1D4-BACE1-HEK293 cells were treated for 16 hours in the absence (control, white circles) or in the presence of WNF (100μg/ml in DMEM/1% FBS, black circles). Cells were then assayed for their β-secretase activity. Values in curves represent the means ± SE of the specific (JMV1197-sensitive) fluorescence recorded during 3 independent experiments. ns, non-statistically different. (F) Cultured wild-type HEK293 cells were incubated without (control) or with the indicated concentrations of WNF (in 1ml DMEM/1% FBS) for 16 hours at 37°C. Cells were then collected and endogenous BACE1 and β-actin were analyzed by Western blot. Immunoblots illustrate representative gels and histograms correspond to the statistical analysis for all experiments. All bars correspond to the densitometry analyses (BACE1 normalized with β-actin), are expressed as a percentage of control (white bars, non treated cells) taken as 100 and are the means ± SE of 4 independent experiments. ns, non-statistically different.

RETRACTED

We next examined the ability of WNF to stimulate sAPPα production in the previously well-characterized MEFs derived from wild-type, ADAM10^-/-^ and ADAM17^-/-^ animals [20–22]. Because the anti-sAPPα antibody DE2B4 is human-specific, we transiently transfected human βAPP_751_. As shown in Fig 4A and 4B, the three cell lines efficiently overexpressed human βAPP and secreted detectable amounts of human sAPPα at 36 hours post-transfection. Importantly, WNF (100μg/ml) could promote the constitutive (Fig 4A, upper left panel) and PKC-regulated (Fig 4B, upper left panel) release of sAPPα in the wild-type MEFs, but not in ADAM10 and ADAM17 knockout cells respectively (Fig 4A and 4B, upper right panels). Moreover, the positive effects of WNF toward both the constitutive (Fig 4C, left panel) and PDBu-induced (Fig 4D, left panel) JMV2770-hydrolyzing activities observed in wild-type MEFs were fully prevented by ADAM10 (Fig 4C, right panel) and ADAM17 depletions (Fig 4D, right panel) respectively. Altogether, these data undoubtedly established ADAM10 and ADAM17 as genuine mediators of WNF-dependent α-secretase activation.

**Fig 4:** ADAM10 and ADAM17 knockouts respectively abolish the constitutive and PDBu-stimulated WNF-induced sAPPα secretions and JMV2770 hydrolysis in mouse embryonic fibroblasts. (A, B) Wild-type (WT) (A, B, left panels), ADAM10^-/-^ (A, right panel) or ADAM17^-/-^ (B, right panel) MEFs were transfected for 24 hours with empty or human βAPP_751_-encoding pcDNA3. Eight hours post transfection, cells were incubated without (-) or with (+) WNF (100μg/ml) for 16 hours (in 1ml of DMEM/1% FBS). Cells in (B) were subsequently treated with PDBu (1μM) for 2 hours and all cells were allowed to secrete for 3 hours (in 1ml serum-free DMEM). Proteins in media were precipitated with 15% TCA and cells were collected and homogenized in lysis buffer. sAPPα, βAPP and β-actin were detected by western blot. (C, D) Wild-type (WT) (C, D, left panels), ADAM10^-/-^ (C, right panel) or ADAM17^-/-^ (D, right panel) MEFs were incubated without (CT) or with WNF (100μg/ml) for 16 hours (in 1ml of DMEM/1% FBS). Cells in (D) were subsequently treated with PDBu (1μM) for 2 hours. JMV2770 (10μM) was then added (in 1.5 ml of PBS) in the absence or in the presence of o-phenanthroline (100μM) and fluorescence was recorded. Values in black bars are expressed as the percent of control (no treatment, white bars) calculated at 30 min and are the means ± SE of 6 to 10 independent experiments. *p<0.03; **p<0.02; ns, non-statistically different.

RETRACTED

To determine whether WNF up-regulates ADAM10 and ADAM17 expressions, we first measured the impact of WNF treatment on ADAM10 and ADAM17 protein levels in HEK293 cells by western blot. Surprisingly, WNF (100μg/ml) significantly increased ADAM10 (Fig 5A, left panels) but not ADAM17 endogenous immunoreactivities (Fig 5A, right panels). We next performed quantitative real-time PCR experiments and established that WNF treatment leads to a significant augmentation of ADAM10 but not ADAM17 mRNA levels (Fig 5B). Because WNF apparently triggers ADAM17 maturation as illustrated by an increase of active ADAM17 (lower band, Fig 5A upper right panel), velocity sedimentation of ADAM10 and ADAM17 in sucrose step gradients was performed. Partial characterization of the fractions, using anti-58K Golgi protein and anti-calnexin antibodies as markers of the Golgi apparatus and the endoplasmic reticulum (ER), indicated that these organelles reside in fractions 1–3 and fractions 11–12 respectively (Fig 5C panels e and f). The results indicated that whereas the distribution profiles of endogenous ADAM10 was similar in control and WNF-treated cells (Fig 5C panels a and b), the maturation of endogenous ADAM17 was strongly enhanced by WNF, thereby increasing ADAM17 maturation in the Golgi/trans-Golgi network (TGN) (compare mature ADAM17 immunoreactivity in fractions 1–3 for panels c and d in Fig 5C) as well as the level of active ADAM17 in the ER/plasma membrane fractions (Fig 5C, lanes 11 and 12 in panels c and d).

**Fig 5:** WNF up-regulates ADAM10 and ADAM17 via two distinct mechanisms in human HEK293 cells. (A, B) HEK293 cells were treated for 36 hours without (control) or with WNF (100μg/ml) in DMEM/1% FBS. (A) ADAM10 (left panel), ADAM17 (right panel) as well as β-actin immunoreactivities were assayed by western blot. (B) ADAM10, ADAM17 as well as GAPDH mRNA levels were determined by real-time PCR. Black bars in histograms correspond to the densitometric analyses normalized with β-actin (A) or mRNA levels normalized with GAPDH (B), are expressed as a percentage of control (non-treated cells, white bars) and represent the means ± SE of 11 to 17 independent determinations. *p<0.0005; **p<0.0001; ns, non-statistically different. (C) HEK293 were incubated for 16 hours without (control) or with WNF (100μg/ml), homogenized and the sub-cellular distributions of endogenous ADAM10 (panels a and b), ADAM17 (panels c and d) as well as the ER marker calnexin (panel e) and the Golgi marker Golgi 58K protein (panel f) were analyzed by western blot after sucrose gradient fractionation. TGN, trans-golgi network; ER/PM, endoplasmic reticulum/plasma membrane.

RETRACTED

Finally, because α-secretase cleaves βAPP in the middle of the Aβ sequence, we hypothesized that WNF treatment could affect amyloid peptides generation in non-neuronal and neuronal human cells transiently overexpressing human βAPP. Firstly, thirty-six hours post-transfection, both HEK293 and SH-SY5Y cells express high βAPP levels when compared to pcDNA3-transfected cells (Fig 6A and 6B upper panels). Secondly and remarkably, WNF applied at a dose of 100μg/ml significantly reduced the secretion of Aβ40 as well as the toxic and aggregate-prone Aβ42 peptide in HEK293 cells (Fig 6A) as well as in the SH-SY5Y neuroblastoma cell line (Fig 6B).

**Fig 6:** WNF decreases Aβ peptides generation in HEK293 and SH-SY5Y human cells. HEK293 (A) and SH-SY5Y cells (B) transiently transfected with human wild-type βAPP_751_ for 36 hours were incubated in the absence (white bars) or in the presence (black bars) of WNF (100μg/ml) during the last 16 hours in 600μl of DMEM/1% FBS. Proper βAPP overexpression was assessed by western blot (upper panels) and human Aβ40 and Aβ42 were measured in 50μl of the 16 hours-secretion media by ELISA. Data are presented after normalization to βAPP and β-actin, values in black bars are expressed as the percent of control (no treatment, white bars) and are the means ± SE of 6 independent determinations. *p<0.02; **p<0.0001.

## Discussion

Together with Aβ-targeting vaccination, the pharmacological inhibition of the two β- and γ-secretases Aβ-forming enzymes stood during the past decades as the principal and most relevant therapeutic tracks aimed at preventing, slowing down or curing Alzheimer’s disease. However, because BACE1 and γ-secretase cleave, in addition to βAPP, a constantly growing number of other substrates with important physiological functions, this strategy may engender severe deleterious side effects. Considering this matter of fact, a more recently developed alternative consists in the activation of the α-secretases ADAM10 and ADAM17. The principal advantage of such an approach as an anti-AD therapy resides in the fact that stimulation of this cleavage is not only expected to preclude Aβ production but also to support neurotrophism, neuroprotection and neurogenesis through an increased secretion of the βAPP-derived sAPPα metabolite. Unfortunately, because ADAM10 and/or ADAM17 have more than 80 other substrates, the cleavages of which yielding to pathological situations such as cancer and chronic inflammation [9], one should stay very cautious regarding the use of acute pharmacological activation of α-secretases and to rather envision stimulating these proteases via the mild, safe and regular consumption of natural compounds that would reduce the amyloid load on a long term basis and could thereby represent a valuable therapeutic alternative for AD treatment [26].

RETRACTED

Falling within such an approach, the present study proposed to investigate the effect of the polyherbal Wattana formula on the non-amyloidogenic processing of βAPP *in vitro* in various cell lines by means of complementary techniques aimed at measuring sAPPα secretion, Aβ production as well as α-secretase catalytic activities, expression and subcellular distribution. We first established that WNF stimulates the constitutive and the PKC-regulated α-secretase activities in a dose-dependent manner. Importantly, WNF not only stimulates sAPPα secretion in βAPP-overexpressing non-neuronal HEK293 and neuroblastoma N2a cells, thereby indicating its ubiquitous action, but also behaves as a potent enhancer of endogenous sAPPα production in the human SH-SY5Y neuroblastoma cell line. In addition, using pharmacological inhibition and genetic depletion approaches, we formally identified ADAM10 and ADAM17 as the targeted proteases, thereby establishing WNF as a potent α-secretase enhancer and a possible anti-AD agent. It is important to underline here that, as far as the amyloid cascade hypothesis is considered to be at the center of gravity of the pathology, α-secretase natural activators in general and WNF in particular are expected to bring preventive rather than curative beneficial effects since they theoretically impair all the following events such as Aβ oligomerization and fibrillogenesis as well as the subsequent cognitive impairments associated with the disease.

Our observations that WNF does not interfere with the amyloidogenic β-secretase activity but significantly lowers both Aβ40 and Aβ42 production underline the fact that any therapeutic strategy leading to α-secretase activation with no modification of β-secretase activity is expected to be sufficient to impair Aβ generation and is in good agreement with the observation that the sole ADAM10 overexpression reduces both Aβ40 and Aβ42 levels *in vivo* in the brain of a transgenic mouse model of AD [27].

On a mechanistic point of view, it is of utmost interest to underline that ADAM10 and ADAM17, although presenting a similar general structure, are up-regulated by WNF via two distinct mechanisms. Thus, WNF induces an elevation of ADAM10 immunoreactivity and mRNA levels thereby demonstrating an effect at the transcriptional level. However, the same treatment has no impact on ADAM17 transcription but rather promotes its maturation/activation as shown by the marked increase of active ADAM17 and the concomitant decrease of the pro-enzyme (Fig 4C, bottom panels). Because WNF is a mixture of 15 medicinal plants, the most probable explanation would be that ADAM10 and ADAM17 are targeted by distinct WNF components, the identification of which remaining to be established.

RETRACTED

In this respect, some of the molecules identified as part of the WNF by ultra-performance liquid chromatography [14] were indeed recently shown to be beneficial regarding AD pathology. Firstly, the active alkaloid and acetylcholinesterase inhibitor piperine can protect against neurodegeneration and cognitive impairment in a rat model of AD [28]. Secondly, the antioxidant and anti-inflammatory polyphenol gallic acid is able to decrease Aβ toxicity [29], to reduce amyloid fibril formation [30] and to attenuate neuronal damage by preventing Aβ oligomerization [31]. Thirdly, the antioxidant and NFκB inhibitor p-coumaric acid as well as the phenolic compound caffeic acid protect against Aβ25–35-induced neurotoxicity respectively *in vitro* in PC12 cells [32] and *in vivo* in rats [33]. Fourthly, ferulic acid, a phenol that is closely related to curcumin and has antioxidant properties, induces a resistance to Aβ42 toxicity in adult mice [34] and reduces amyloid deposition in a mouse model of AD [35]. However, contrary to our findings, all these described effects most likely occur at a late post-Aβ production step rather than at earlier βAPP processing stages. Nevertheless, two recent publications have evidenced that some of these compounds can indeed target βAPP-cleaving secretases. Hence, ferulic acid can reverse the behavioral deficits of the PSAPP transgenic mouse model of AD through a slight reduction of the β-secretase BACE1 stability and activity [36] that we could not detect in the whole extract. Moreover, octyl gallate, the ester of 1-octanol and gallic acid, has been shown to inhibit Aβ generation and to increase sAPPα secretion *in vitro* and *in vivo* via an increase of estrogen receptor-mediated ADAM10 activity [37] and could therefore support the WNF-dependent increase of ADAM10 activity/expression observed in the present study.

It is also worth mentioning that besides its herein described α-secretase-stimulating property, WNF may also provide an additional and complementary beneficial anti-AD effect since five of its components (*Aucklandialappa* DC. (Costus); *Terminalia chebula* Retz. (Myrobalans); *Piper nigrum* L. (White Pepper); *Cyperusrotundus* L. (Nutgrass) and *Aegle marmelos* (L.) Corrêa (Bael fruit)) display acetylcholinesterase inhibitory activity [38–40].

RETRACTED

Supporting the promising anti-AD therapeutic use of medicinal plants, several other plant extracts have been recently reported to convey beneficial effects in *vivo* in animal models of AD ([41] for review). Firstly, extracts prepared from *Centella asiatica* (L.) Urb. (Umbelliferae) were shown to ameliorate cognitive performances and to decrease Aβ levels, oxidative stress and senile plaques formation [42, 43]. Secondly, extract from *Bacopa monnieri* (L.) Wettst. (Brahmi) displays neuroprotective effects, reduces Aβ production and can improve cognitive functions [44, 45]. Finally, extracts from *Withania somnifera* (L.) Dunal diminish behavioral deficits, Aβ production and plaque pathology [46]. Following the present demonstration that WNF is able to increase sAPPα secretion and to reduce Aβ production *in vitro*, evaluating whether individuals who regularly consume WNF are less prone to developing AD will be of particular interest.

## Conclusion

This study clearly establishes WNF as a potent *in vitro* activator of the non-amyloidogenic processing of βAPP. Because this is accompanied by a reduction of amyloid peptides production, it is our assumption that WNF may be used as a mild natural anti-AD preventive treatment. The identification of the WNF-containing active molecule(s) as well as the demonstration that WNF can slow down or reverse the pathology in transgenic mouse models of AD should deserve a particular attention in a near future. However, it is important to underline here that, regardless of this considerations, the use of this polyherbal formula is already possible for further clinical studies in humans since it is currently prescribed to patients for the treatments of AD-unrelated symptoms and does not display any secondary effects.

## References

[1] ZhangH, MaQ, ZhangYW, XuH. Proteolytic processing of Alzheimer’s β-amyloid precursor protein. J Neurochem. 2012;120(Suppl.1):9–21.2212237210.1111/j.1471-4159.2011.07519.xPMC3254787

[2] MattsonMP, ChengB, CulwellAR, EschFS, LieberburgI, RydelRE. Evidence for excitoprotective and intraneuronal calcium-regulating roles for secreted forms of the β-amyloid precursor protein. Neuron 1993;10:243–254. 809496310.1016/0896-6273(93)90315-i

[3] FurukawaK, SopherBL, RydelRE, BegleyJG, PhamDG, MartinGM, et al Increased activity-regulating and neuroprotective efficacy of α-secretase-derived secreted amyloid precursor protein conferred by a C-terminal heparin-binding domain. J Neurochem. 1996;67(5):1882–1896. 886349310.1046/j.1471-4159.1996.67051882.x

RETRACTED

[4] ClaasenAM, GuévremontD, Mason-ParkerSE, BourneK, TateWP, AbrahamWC, et al Secreted amyloid precursor protein-α upregulates synaptic protein synthesis by a protein kinase G-dependent mechanism. Neurosci Lett. 2009;460:92–96. 10.1016/j.neulet.2009.05.040 19463893

[5] MezianeH, DodartJC, MathisC, LittleS, ClemensJ, PaulSM, et al Memory-enhancing effects of secreted forms of the β-amyloid precursor protein in normal and amnestic mice. Proc Natl Acad Sci USA 1998;95:12683–12688. 977054610.1073/pnas.95.21.12683PMC22891

[6] CailléI, AllinquantB, DupontE, BouillotC, LangerA, MullerU, et al Soluble form of amyloid precursor protein regulates proliferation of progenitors in the adult subventricular zone. Development 2004;131(9):2173–2181. 10.1242/dev.01103 15073156

[7] VincentB, GovitrapongP. Activation of the α-secretase processing of AβPP as a therapeutic approach in Alzheimer’s disease. J Alzheimers Dis. 2011;24(Suppl.2):75–94.2142251510.3233/JAD-2011-110218

[8] WooHN, BaikSH, ParkJS, GwonAR, YangS, YunYK, et al Secretases as therapeutic targets for Alzheimer’s disease. Biochem Biophys Res Commun. 2011;404(1):10–15. 10.1016/j.bbrc.2010.11.132 21130746

[9] VincentB, CheclerF. α-secretase in Alzheimer’s disease and beyond: mechanistic, regulation and function in the shedding of membrane proteins. Curr Alzheimer Res. 2012;9(2):140–56. 2160503110.2174/156720512799361646

[10] WollenKA. Alzheimer’s disease: the pros and cons of pharmaceuticals, nutritional, botanical, and stimulatory therapies, with a discussion of treatment strategies from the perspective of patients and practitioners. Altern Med Rev. 2010;15(3):223–44. 21155625

[11] PanichU, PluemsamranT, Tangsupa-a-nanV, WattanarangsanJ, PhadungrakwittayaR, AkarasereenontP, et al Protective effect of AVS073, a polyherbal formula, against UVA-induced melanogenesis through a redox mechanism involving glutathione-related antioxidant defense. BMC Complement Altern Med. 2013;13:159 10.1186/1472-6882-13-159 23826868PMC3706233

[12] BunnanK, ChaikominR, LohsiriwatS, ChomchaiS, AkarasereenontP. Effect of Ayuraved Siriraj herbal recipe “Wattana” on gastric emptying rate. Siriraj Med J. 2012;64(3):89–93.

[13] PengkhumT, ChatsiricharoenkulS, AkarasereenontP, CharoencholvanichK. Phase II clinical trial of Ayurved Siriraj Wattana recipe for symptomatic relief in patients with osteoarthritis of the knee. J Med Assoc Thai. 2012;95(3):452–60. 22550847

[14] Duangsa-ardS, WongkajornsilpA, AkarasereenontP, HuabprasertS, ChongputtharaksaT, LaohapandT. The effects of Ayurved Siriraj Wattana recipe on splenocytes in Wistar rat. Siriraj Med J. 2013;65(3):73–6.

RETRACTED

[15] WongkajornsilpA, NumchaisermsukN, Sa-ngiamsuntornK, AkarasereenontP, WamanuttajindaV, KasetsinsombatK, et al Effects of the Ayurved Siriraj Wattana recipe on functional and phenotypic characterization of cytokine-induced killer cells and dendritic cells in vitro. BMC Complement Altern Med. 2016;16:489 10.1186/s12906-016-1480-7 27899095PMC5129228

[16] AndrauD, Dumanchin-NjockC, AyralE, VizzavonaJ, FarzanM, BoisbrunM, et al BACE1- and BACE2-expressing human cells. Characterization of β-amyloid precursor protein-derived catabolites, design of a novel fluorimetric assay, and identification of new *in vitro* inhibitors. J Biol Chem. 2003;278(28):25859–66. 10.1074/jbc.M302622200 12736275

[17] MarambaudP, ChevallierN, BarelliH, WilkS, CheclerF. Proteasome contributes to the α-secretase pathway of amyloid precursor protein in human cells. J Neurochem. 1997;68(2):698–703. 900305810.1046/j.1471-4159.1997.68020698.x

[18] VincentB, PaitelE, FrobertY, LehmannS, GrassiJ, CheclerF. Phorbol ester-regulated cleavage of normal prion protein in HEK293 human cells and murine neurons. J Biol Chem. 2000;275(45):35612–16. 10.1074/jbc.M004628200 10952979

[19] BorcheltDR, ThinakaranG, EckmanCB, LeeMK, DavenportF, RatovitskyT, et al Familial Alzheimer’s disease-linked presenilin 1 variants elevate Aβ1-42/1-40 ratio in vitro and in vivo. Neuron 1996;17(5):1005–13. 893813110.1016/s0896-6273(00)80230-5

[20] BlackRA, RauchCT, KozloskyCJ, PeschonJJ, SlackJL, WolfsonMF, et al A metalloproteinase disintegrin that releases tumour-necrosis factor-α from cells. Nature 1997;385(6618):729–33. 10.1038/385729a0 9034190

[21] HartmannD, de StrooperB, SerneelsL, CraessaertsK, HerremanA, AnnaertW, et al The disintegrin/metalloprotease ADAM10 is essential for notch signaling but not for α-secretase activity in fibroblasts. Hum Mol Genet. 2002;11(21):2615–24. 1235478710.1093/hmg/11.21.2615

[22] ShuklaM, HtooHH, WintachaiP, HernandezJF, DuboisC, PostinaR, et al Melatonin stimulates the nonamyloidogenic processing of βAPP through the positive transcriptional activation of ADAM10 and ADAM17. J Pineal Res. 2015;58(2):151–65. 10.1111/jpi.12200 25491598

[23] BradfordMM. A rapid and sensitive method for the quantification of microgram quantities of protein utilizing the principle of protein-dye binding. *Anal*. *Biochem*. 1976;72:248–54. 94205110.1016/0003-2697(76)90527-3

[24] Alfa CisséM, GandreuilC, HernandezJF, MartinezJ, CheclerF, VincentB. Design and characterization of a novel cellular prion-derived quenched fluorimetric substrate of α-secretase. Biochem Biophys Res Commun. 2006;347(1):254–60. 10.1016/j.bbrc.2006.06.065 16806063

[25] VingtdeuxV, MarambaudP. Identification and biology of α-secretase. J Neurochem. 2012;120(Suppl.1):34–45.2212187910.1111/j.1471-4159.2011.07477.x

RETRACTED

[26] EssaMM, VijayanRK, Castellano-GonzalezG, MemonMA, BraidyN, GuilleminGJ. Neuroprotective effect of natural products against Alzheimer’s disease. Neurochem Res. 2012;37(9):1829–42. 10.1007/s11064-012-0799-9 22614926

[27] PostinaR, SchroederA, DewachterI, BohlJ, SchmittU, KojroE, et al A disintegrin-metalloproteinase prevents amyloid plaque formation and hippocampal defects in an Alzheimer disease mouse model. J Clin Invest. 2004;113(10):1456–64. 10.1172/JCI20864 15146243PMC406531

[28] ChonpathompikunlertP, WattanathornJ, MuchimapuraS. Piperine, the main alkaloid of Thai black pepper, protects against neurodegeneration and cognitive impairment in animal model of cognitive deficit like condition of Alzheimer’s disease. Food Chem Toxicol. 2010;48(3):798–802. 10.1016/j.fct.2009.12.009 20034530

[29] KimMJ, SeongAR, YooJY, JinCH, LeeYH, KimYJ, et al Gallic acid, a histone acetyltransferase inhibitor, suppresses β-amyloid neurotoxicity by inhibiting microglial-mediated neuroinflammation. Mol Nutr Food Res. 2011;55(12):1798–1808. 10.1002/mnfr.201100262 22038937

[30] LiuY, PukalaTL, MusgraveIF, WilliamsDM, DehleFC, CarverJA. Gallic acid is the major component of grape seed extract that inhibits amyloid fibril formation. Bioorg Med Chem Lett. 2013;23(23):6336–40. 10.1016/j.bmcl.2013.09.071 24157371

[31] HajipourS, SarkakiA, FarboodY, EidiA, MortazaviP, ValizadehZ. Effect of gallic acid on dementia type of Alzheimer’s disease in rats: electrophysiological and histological studies. Basic Clin Neurosci. 2016;7(2):97–106. 10.15412/J.BCN.03070203 27303604PMC4892325

[32] YoonJH, YounK, HoCT, KarweMV, JeongWS, JunM. *p*-coumaric acid and ursolic acid from *Corni fructus* attenuated β-amyloid_25-35_-induced toxicity through regulation of the NFκB signaling pathway in PC12 cells. J Agric Food Chem. 2014;62(21):4911–16. 10.1021/jf501314g 24815946

[33] KimJH, WangQ, ChoiJM, LeeS, ChoEJ. Protective role of caffeic acid in an Aβ_25-35_-induced Alzheimer’s disease model. Nutr Res Pract. 2015;9(5):480–8. 10.4162/nrp.2015.9.5.480 26425277PMC4575960

[34] YanJJ, ChoJY, KimHS, KimKL, JungJS, HuhSO, et al Protection against β-amyloid peptide toxicity *in vivo* with long-term administration of ferulic acid. Brit J Pharmacol. 2001;133(1):89–96.1132579810.1038/sj.bjp.0704047PMC1572763

[35] YanJJ, JungJS, KimTK, HasanMA, HongCW, NamJS, et al Protective effects of ferulic acid in amyloid precursor protein plus presenilin-1 transgenic mouse model of Alzheimer’s disease. Biol Pharm Bull. 2013;36(1):140–3. 2307567810.1248/bpb.b12-00798

[36] MoriT, KoyamaN, Guillot-SestierMV, TanJ, TownT. Ferulic acid is a nutriceutical β-secretase modulator that improves behavioral impairment and Alzheimer-like pathology in transgenic mice. PLoS ONE 2013;8(2):e55774 10.1371/journal.pone.0055774 23409038PMC3568151

RETRACTED

[37] ZhangSQ, SawmillerD, LiS, Rezai-ZadehK, HouH, ZhouS, et al Octyl gallate markedly promotes anti-amyloidogenic processing of APP through estrogen receptor-mediated ADAM10 activation. PLoS ONE 2013;8(8):e71913 10.1371/journal.pone.0071913 23977176PMC3744472

[38] IngkaninanK, TemkitthawonP, ChuenchomK, YuyaemT, ThongnoiW. Screening for acetylcholinesterase inhibitory activity in plants in Thai traditional rejuvenating and neurotonic remedies. J Ethanopharmacol. 2003;89(2–3):261–4.10.1016/j.jep.2003.08.00814611889

[39] AsaduzzamanM, UddinMJ, KaderMA, AlamAHMK, RahmanAA, RashidM, et al In vitro acetylcholinesterase inhibitory activity and the antioxidant properties of *Aegle marmelos* leaf extract: implications for the treatment of Alzheimer’s disease. Psychogeriatrics 2014;14(1):1–10. 10.1111/psyg.12031 24646308

[40] MathewM, SubramanianS. In vitro screening for anti-cholinesterase and antioxidant activity of methanolic extracts of Ayurvedic medicinal plants used for cognitive disorders. PLoS ONE 2014;9(1):e86804 10.1371/journal.pone.0086804 24466247PMC3900633

[41] RaoRV, DescampsO, JohnV, BredesenDE. Ayurvedic medicinal plants for Alzheimer’s disease. Alzheimer’s Res Ther. 2012;4(3):22.2274783910.1186/alzrt125PMC3506936

[42] VeerendraKumar MH, GuptaYK. Effect of *Centella asiatica* on cognition and oxidative stress in an intracerebroventricular streptozotocin model of Alzheimer’s disease in rats. Clin Exp Pharmacol Physiol. 2003;30(5–6):336–42. 1285942310.1046/j.1440-1681.2003.03842.x

[43] DhanasekaranM, HolcombLA, HittAR, TharakanB, PorterJW, YoungKA, et al *Centella asiatica* extract selectively decreases amyloid β levels in hippocampus of Alzheimer’s disease animal model. Phytother Res. 2009;23(1):14–19. 10.1002/ptr.2405 19048607

[44] HolcombLA, DhanasekaranM, HittAR, YoungKA, RiggsM, ManyamBV. *Bacopa monniera* extract reduces amyloid levels in PSAPP mice. J Alzheimers Dis. 2006;9(3):243–51. 1691483410.3233/jad-2006-9303

[45] UabunditN, WattanathornJ, MucimapuraS, IngkaninanK. Cognitive enhancement and neuroprotective effects of *Bacopa monnieri* in Alzheimer’s disease model. J Ethnopharmacol. 2010;127:26–31. 10.1016/j.jep.2009.09.056 19808086

[46] SehgalN, GuptaA, ValliRK, JoshiSD, MillsJT, HamelE, et al *Withania somnifera* reverses Alzheimer’s disease pathology by enhancing low-density lipoprotein receptor-related protein in liver. Proc Natl Acad Sci U.S.A 2012;109(9):3510–5. 10.1073/pnas.1112209109 22308347PMC3295277

